# Different Intestinal Microbiota with Growth Stages of Three-Breed Hybrid Pig

**DOI:** 10.1155/2022/5603451

**Published:** 2022-08-08

**Authors:** Cheng-xing Long, Jie-qi Wu, Zhou-jin Tan, Sheng-ping Wang

**Affiliations:** ^1^Hunan University of Humanities, Science and Technology, Loudi, China; ^2^Loudi Fisheries Science Research Institute, Loudi, China; ^3^Hunan University of Chinese Medicine, Changsha, China; ^4^Hunan Institute of Microbiology, Changsha, China

## Abstract

The changes of intestinal microbiota are closely related to the growth and development of animals. The current study is aimed at exploring the composition of the microbial community of pigs at different growth stages. Fresh fecal samples of three-breed hybrid pigs at three developmental stages (60, 120, and 180 days of age) were collected. The microbial composition was analyzed based on the 16S rDNA gene of bacteria Illumina NovaSeq sequencing platform. The results showed that the intestinal microbiota of pigs was distributed in 22 phyla, 46 classes, 84 orders, 147 families, and 287 genera. Firmicutes, Bacteroides, Spirochaetae, Proteobacteria, and Actinobacteria were the dominant phyla. *Lactobacillus*, *Streptococcus*, *SMB*53, *Oscillospira*, and *Prevotella* were the dominant genera. Among them, the abundance of *Lactobacillus* and *SMB*53 increased first and then decreased, while the change of *Oscillospira* was opposite. In addition, the abundance of *Streptococcus* increased while that of *Prevotella* decreased gradually. Moreover, with the increase of time and body weight, the microbial diversity showed a decreasing trend. In conclusion, the intestinal microbial composition of the three-breed hybrid pigs was relatively stable during the fattening stage, but there were significant differences in abundance.

## 1. Introduction

Pig intestinal microbiota is a complex microecosystem, mainly composed of anaerobic bacteria and facultative anaerobic bacteria, among which Firmicutes and Bacteroidetes are the dominant bacteria accounting for more than 90%, playing an important role in maintaining body health, and improving body immunity, nutrient absorption, and metabolism [1]. Under the influence of factors such as strain [2–4], age [5, 6], diet [7–10], environment [11], and pathogen microbial infection [12], the intestinal microbiota of pigs presents dynamic structure and diversity. There are significant differences in the intestinal microbiota of pigs at different stages, and the intestinal microbiota structure of pigs is basically formed within 2-3 weeks after weaning. After that, growth and development and dietary changes are the main causes of continuous changes in the intestinal microbiota structure of pigs [13, 14]. Although there have been many studies on the intestinal microbiota of pigs at different stages, there have been no reports on the characteristics of the intestinal microbiota of three-breed hybrid pigs during growing and fattening periods.

It is well known that there are abundant pig breed resources in China, and some of which have strong growth performance and reproductive capacity [15, 16]. However, there are significant differences in various indexes of pigs among different breeds [17, 18]. Three-breed hybrid pig, also known as “Duroc×Landrace×Yorkshine,” is bred from Duroc and Landrace as parents. It is one of the excellent hybrid breeds in China and also one of the largest pig breeds nowadays because of its medium in size, early maturity, easy to fat, good meat quality, and strong resistance [19, 20].

In this study, samples of three-hybrid pigs were provided by Yiyou Ecological Breeding Co., Ltd., Lianyuan City, Hunan Province. The dynamic changes of intestinal microbiota in different growth and fattening period of pigs were analyzed using 16S rRNA sequencing technology and bioinformatics methods to reveal the composition characteristics of intestinal microbes in different pig breeds at different growth stages. These results will provide a reference for improving the microbial basis of pig growth performance and health.

## 2. Materials and Methods

### 2.1. Selection of Experimental Pigs

Healthy pigs with the same batch, the same age, and the same body weight were selected under identical husbandry practices and epidemic prevention systems in Yiyou Ecological Breeding Co., Ltd., Lianyuan City, Hunan Province. Pigs were raised on solid feed (Xiang Feeding Certificate (2015) 04063). The diet provided crude protein (≥16.5%), crude fiber (≤7.0%), crude ash (≤8.0%), calcium (0.5%-1.2%), total phosphorus (≥0.4%), sodium chloride (0.3%-0.8%), lysine (≥1.05%), and moisture (≤1.05%). Fresh feces samples of pigs were collected at three stages (60 days, 180 days, and 180 days of age) directly using sterile tools or sterile cotton swabs. All procedures involving animals were performed according to protocols approved by the Institutional Animal Care and Use Committee of Hunan University of Chinese Medicine (No. 20171202).

### 2.2. Sample Collection and Preservation

There were five pigs in each group. The average body weights of pigs in three groups were 154.592 ± 4.245 kg (180 days group, SM), 102.416 ± 2.379 kg (120 days group, FM), and 29.386 ± 0.513 kg (60 days group, TM), respectively. The fresh fecal samples were collected from the same pig farm on September 13, 2020 in Lianyuan, Hunan, China (111.67 N; 27.69 W). Sealed in dry ice and immediately brought back to the laboratory for storage at -80°C.

### 2.3. DNA Extraction and PCR Amplification

DNA was extracted from the retained content samples following the instructions of the extraction kit. The purity and concentration of extracted DNA samples were detected by ultraviolet spectrophotometer [21]. The integrity of samples was detected by gel electrophoresis. The qualified samples were amplified by Shanghai Personal Biotechnology Co., Ltd. (Shanghai, China). 16S rRNA gene primers 338F: 5′-ACTCCTACGGGAGGCAGCA-3′ and 806R: 5′-GGACTACHVGGGTWTCTAAT-3′ were used for PCR amplification of V3-V4 region of bacterial 16S rRNA gene. Reaction system is as follows: (25 *μ*L):5 × reaction buffer 5 *μ*L, 5 × GC buffer 5 *μ*L, dNTPs (2.5 mM) 2 *μ*L, forwardprimer (10 *μ*M) 1 *μ*L, reverseprimer (10 *μ*M) 1 *μ*L, DNA template 2 *μ*L, ddH2O 8.75 *μ*L, and Q5 DNA polymerase 0.25 *μ*L. Amplification parameters are as follows: initial denaturation 98°C 2 min, denaturation 98°C 15 s, rolling at 55°C 30 s, extension 72°C 30 s, final Extension 72°C 5 min, and 10°C hold 25 to 30 cycles.

### 2.4. Illumina NovaSeq Sequencing

Each sample contained 5 replicates. PCR products of the same sample were mixed and detected by 2% agarose gel electrophoresis. Sequencing was performed using the Illumina NovaSeq platform under Illumina's standard procedure (Illumina, San Diego, CA, USA). Sequencing was performed by Shanghai Personal Biotechnology Co., Ltd. (Shanghai, China).

### 2.5. Sequence Optimization and OTU Clustering

The Vsesion7.1 software in Usearch platform was used to perform OTU (Operational Taxonomic Unit) cluster analysis for the sequences after quality control [22]. The QIIME2 software (http://github.com/QIIME2/q2-feature-classifier) was used for quality control, filtering, and decontamination of the original data obtained from sequencing, and OTU clustering of nonrepeating sequences was performed according to 97% similarity [23]. The obtained OTU was classified and identified at different classification levels based on Greengenes database (Release 13.8, http://greengenes.second-genome.com/) [24, 25].

### 2.6. Diversity Analysis

Alpha diversity represents species within-habitat diversity, and beta diversity represents species between-habitat diversity. Both of them are helpful to evaluate the overall diversity of species comprehensively [26, 27]. Chao1 index and Observed Species index represent the richness [28], and the larger the Chao1 and Observed Species indexes, the higher the richness of the community. Shannon index and Simpson index represent diversity [29–31], and the larger the Shannon and Simpson indexes, the higher community diversity. Good's coverage index represents coverage [32], and the higher the Good's coverage index, the lower the proportion of undetected species in the sample. The beta diversity index focuses on the comparison of diversity between different habitats. It was characterized by principal coordinate analysis (PCoA) [33, 34] and nonmetric multidimensional scale analysis (NMDS) [35], aiming to reduce the dimension decomposition of the sample distance matrix, reflect the distance relationship of the original sample, and reveal the differences between samples. The QIIME software (2019.4) was used to calculate Chao1 index, Observed Species index, Shannon index, and Simpson index and analyze PCoA and NMDS.

### 2.7. Species Difference Analysis and Marker Species

LEfSe is an analytical method based on linear discriminant analysis (LDA) effect size. Its essence is to screen key biomarkers by combining linear discriminant analysis with nonparametric Kruskal-Wallis and Wilcoxon rank-sum test [36].

### 2.8. Statistical Analysis

SPSS24.0 statistical software was used for data statistics. A one-way analysis of variance was used for differences among normal distribution data groups, and Mann-Whitney *U* test was used for nonnormal distribution data. Measurement data were expressed as mean ± standard deviation. *P* < 0.05 indicates significant difference, and *P* < 0.01 indicates extremely significant difference. The original sequence obtained in this study has been submitted to the NCBI Sequence Read Archive (accession number is SRP: PRJNA795214, htttp://http://www.ncbi.nlm.nih.gov/).

## 3. Results

### 3.1. Description of Sequencing Data

To observe the microbiota of three-breed hybrid pigs at different growth and development stages, the V3-V4 region of bacterial 16S rDNA genes was sequenced using Illumina NovaSeq platform. After quality control of the measured data, a total of 885695 high-quality sequences were obtained from 15 samples in the three groups, and the dominant sequence lengths were mainly 404-411 bp (47.15%) and 423-432 bp (52.63%) (Figure 1(a)). The average value of Good's coverage index in all samples was 0.9859, between 0.9793 and 0.9912, reflecting the real situation of species in the community (Table 1). As shown in the Venn diagram, a total of 14470 OTUs were obtained in the three groups. There are 6547 in the TM group, accounting for 45.25%. There are 5440 in the FM group, accounting for 37.60%. And there are 4387 in the SM group, accounting for 30.32%. Among them, 952 were identical, accounting for 6.58% (Figure 1(b)). The results showed that the species of intestinal microbiota in three-breed hybrid pigs was inversely proportional to time during fattening.

### 3.2. Diversity of Intestinal Microbiota in Pigs

The QIIME software (2019.4) was used to calculate Chao1 index, Observed Species index, Shannon index, and Simpson index of the samples, and *t*-test analysis was conducted on diversity index of different groups (Figure 2 and Table 1). The variation trend of Chao1 index, Observed Species index, Shannon index, and Simpson index was basically the same, among which Chao1 and Observed Species indexes were significant, indicating that with the increase of pig weight and feeding time, the intestinal microbial diversity of pigs showed a decreasing trend, and the longer the feeding time and the heavier the weight, the lower the decrease and tended to be stable.

### 3.3. Composition of Intestinal Microbiota in Pigs at Different Taxonomic Levels

The microbiota of all samples was counted according to the abundance of species. A total of 22 phyla were detected, among which Firmicutes, Bacteroidetes, Spirochaetes, Proteobacteria, and Actinobacteria were the dominant phyla. At phylum level, Firmicutes increased first and then decreased, increased from 78.73% at 60 days of age to 83.91% at 120 days of age and then decreased to 82.51% at 180 days of age. Bacteroidetes gradually decreased from 16.33% at 60 days of age to 12.11% at 120 days of age and then to 7.29% at 180 days of age. Spirochaetes and Proteobacteria decreased firstly and then increased, from 2.21% and 0.89% at 60 days of age to 0.79% and 0.59% at 120 days of age, and increased to 3.81% and 3.16% at 180 days of age. Actinobacteria increased gradually from 0.35% at 60 days of age to 2.08% at 180 days of age (Figure 3(a) and Table 2).

At the genus level, among the detected bacteria, the top 10 genera in relative abundance were *Lactobacillus*, *Streptococcus*, *SMB*53, *Oscillospira*, *Prevotella*, *Treponema*, *Roseburia*, *Gemmiger*, *Ruminococcus*, and *Clostridiaceae Clostridium*, in which six genera were significantly different (*P* < 0.01 or *P* < 0.05). Among them, *Lactobacillus*, *Streptococcus*, *SMB*53, *Oscillospira*, and *Prevotella* were the dominant genera. *Lactobacillus* and *SMB*53 increased firstly and then decreased, increased from 21.22% and 2.15% at 60 days of age to 25.02% and 8.61% at 120 days of age and then decreased to 11.08% and 5.60% at 180 days of age. *Oscillospira* decreased firstly and then increased, decreased from 6.12% at 60 days of age to 3.05% at 120 days of age and then increased to 3.49% at 180 days of age. *Streptococcus* increased gradually, from 3.44% at 60 days of age to 5.28% at 120 days of age and then to 21.98% at 180 days of age. *Prevotella* decreased gradually, from 5.07% at 60 days of age to 1.83% at 180 days of age (Figure 3(b) and Table 3).

In addition, by PCoA and NMDS analysis (Figures 4(a) and 4(b)), the three groups of samples tended to cluster together, respectively, indicating the relative stability within each sample group. Furthermore, LEfSe analysis showed that *Streptococcaceae* were the biomarkers of the SM group. *SMB* 53 was the biomarker of the FM group. *Oscillospira* was the biomarker in the TM group (Figure 4(c)).

## 4. Discussion

The mammalian gut is a dense, dynamic, and highly complex microbial community with significant differences at different growth stages [37]. Therefore, it is very important to understand the colonization of intestinal microbiota in various growth stages of pigs. The composition of intestinal microbiota of pigs is similar to that of humans, mainly consisting of bacteria, archaea, and eukaryotes, among which the dominant bacteria are anaerobic bacteria such as *Lactobacillus* accounting for more than 99% [38, 39]. At different growth stages, the dominant microbiota in the intestinal tract of pigs has a great relationship with the regulation of autoimmunity. With the increase of age and the change of external environment, the dominant microtiota in the intestinal tract also changes correspondingly, but mainly Firmicutes and Bacteroides [40].

In this study, in order to exclude the effects of feed on intestinal microbiota, pigs were fed with the same feed after weaning. The results showed that the species and abundance of the dominant bacteria in the intestinal tract of pigs at different ages were different, but Firmicutes and Bacteroidetes were the dominant phyla, and the proportion of Firmicutes in the high-age group was higher than that in the low-age group, which was similar to the results of other studies [6]. Firmicutes are the largest and most diverse group of gram-positive bacteria. They mainly participate in the material and energy metabolism of the host and play an extremely important role in the process of food digestion [41]. Bacteroidetes can produce acetate and propionate by fermentation, which can provide necessary substances for host organism and intestinal microorganism [42–44]. Firmicutes and Bacteroidetes are both obesity-related bacteria, and the abundance of Firmicutes is relatively high in obese pigs, while the abundance of Bacteroidetes is relatively low in obese pigs [45].

Intestinal tract is the main site of digestion, absorption, and immune regulation. In this study, the proportion of *Lactobacillus* in the intestinal tract of three-breed hybrid pigs at different ages was the highest, which was closely related to the function of *Lactobacillus* in regulating animal immunity, maintaining bacterial homeostasis and body health, assisting digestion, and improving the growth rate of growing pigs [37, 46]. *Oscillospira* and *Prevotella* are two important short-chain fatty acid-producing bacteria, which can decompose resistant starch and feed fiber and other indigestion substances and produce short-chain fatty acids and other products, playing an important role in energy balance [47, 48]. *Oscillospira* is closely related to body health [49], and *Prevotella* is the main bacteria that mainly digest dietary fiber [50]. Their relatively high abundance is related to the long-term fixed diet after weaning and the crude feeding tolerance of pigs [51, 52]. *Treponema* can produce short-chain fatty acids to regulate the balance of host capacity through fermentation of polysaccharides and glia in the feed [53]. In this study, the abundance of *Treponema* was the highest at 180 days of age, which would be related to the higher crude fiber content in the feed. *Streptococcus*_alactolyticus in *Streptococcus* is a culturable lactic acid bacteria in the jejunum and feces of mammals [54]. *Streptococcus*_alactolyticus was first isolated from the intestinal tract of pigs [55] and was the dominant species in the intestinal tract of pigs [56]. This would be closely related to the growth and reproduction and intestinal health of pigs. In this study, *Streptococcus* occupied a relatively high proportion and had an absolute advantage at 180 days of age, which would be related to the beneficial nature of *Streptococcus*_alactolyticus in *Streptococcus* [57]. The composition and function of these bacteria play an important role in the health level and nutritional value of three-breed hybrid pigs.

There is no doubt that regulating the intestinal microbiota structure can improve the growth efficiency and health level of pigs. Understanding the composition and change process of intestinal microbe during the growth and fattening period of pigs can help prevent the decline of growth performance and health condition caused by intestinal microbe disorder. Our results showed that the composition and structure of intestinal microbiota were relatively stable during the fattening period in three-breed hybrid pigs. But it was still in a state of dynamic change. With the progress of the fattening period, the relative abundance of Firmicutes increased, while that of Bacteroides decreased.

In conclusion, the intestinal microbial compositions of the three-breed hybrid pigs are relatively stable during the fattening stage, but it is still in a state of dynamic change. The results can be used as a reference for constructing a complete database of the three-breed hybrid pig intestinal microbes.

## Figures and Tables

**Figure 1:** Overall description of sequencing data. (a) Sequence length analysis. (b) Venn diagram. TM stands for 60-day group. FM stands for 120-day group. SM stands for 180-day group.

**Figure 2:** Comparison of bacterial alpha diversity analysis. (a) Chao1 index. (b) Observed Species index. (c) Shannon index. (d) Simpson index. TM stands for 60-day group. FM stands for 120-day group. SM stands for 180-day group.

**Figure 3:** Average relative abundance of the on top 10 taxa in each group. (a) At phylum level. (b) At genus level. TM stands for 60-day group. FM stands for 120-day group. SM stands for 180-day group.

**Figure 4:** Comparison of microbial community structure among groups. (a) PCoA. (b) NMDS analysis. (c) LEfSe analysis with LDA score > 4.0. TM stands for 60-day group. FM stands for 120-day group. SM stands for 180-day group.

**Table 1:** Goods coverage and diversity indices of bacterial species during different growth stages.

Group	Chao1	Observed Species	Simpson	Shannon	Goods coverage
TM	2803.01 ± 438.91^∗∗^	2402.62 ± 342.16^∗∗^	0.9743 ± 0.0196	8.4015 ± 0.5467^∗^	0.9834 ± 0.0034^∗^
FM	2493.18 ± 275.45^∗^	2148.06 ± 214.32^∗∗^	0.9638 ± 0.0164	7.8515 ± 0.3439	0.9857 ± 0.0023
SM	1946.21 ± 275.28	1617.18 ± 236.55	0.9329 ± 0.0637	6.9584 ± 0.9996	0.9885 ± 0.0017

Note: TM stands for 60-day group, FM stands for 120-day group, SM stands for 180-day group; compared with SM ^∗^*P* < 0.05 and ^∗∗^*P* < 0.01.

**Table 2:** Main microbiota in different periods at phylum level.

Sample	TM_60 d	FM_120 d	SM_180 d
Firmicutes	0.7873 ± 0.0998	0.8391 ± 0.0719	0.8251 ± 0.1202
Bacteroidetes	0.1633 ± 0.0756	0.1211 ± 0.0687	0.0729 ± 0.0584
Spirochaetes	0.0221 ± 0.0156	0.0079 ± 0.0081	0.0381 ± 0.0364
Proteobacteria	0.0089 ± 0.0134	0.0059 ± 0.0078	0.0316 ± 0.0599
Actinobacteria	0.0035 ± 0.0012^∗^	0.0131 ± 0.0047	0.0208 ± 0.0158
Tenericutes	0.0064 ± 0.0027	0.0074 ± 0.0033	0.0046 ± 0.0026
TM7	0.0047 ± 0.0022^∗^	0.0025 ± 0.0013	0.0023 ± 0.0014
Cyanobacteria	0.0007 ± 0.0005^∗^	0.0013 ± 0.0005	0.0024 ± 0.0020
Verrucomicrobia	0.0008 ± 0.0003^∗∗^	0.0001 ± 0.0001	0.0001 ± 0.0001
Fibrobacteres	0.0005 ± 0.0007	0.0001 ± 0.0001	0.0001 ± 0.0001
Others	0.0018 ± 0.0003	0.0016 ± 0.0007	0.0021 ± 0.0011

Note: TM stands for 60-day group, FM stands for 120-day group, SM stands for 180-day group; compared with SM ^∗^*P* < 0.05 and ^∗∗^*P* < 0.01.

**Table 3:** Main microbiota in different periods at genus level.

Sample	TM_60 d	FM_120 d	SM_180 d
*Lactobacillus*	0.2122 ± 0.1099	0.2502 ± 0.1345	0.1108 ± 0.0675
*Streptococcus*	0.0344 ± 0.0185^∗∗^	0.0528 ± 0.0217^∗∗^	0.2198 ± 0.1382
*SMB*53	0.0215 ± 0.0068	0.0861 ± 0.0522	0.0560 ± 0.0258
*Oscillospira*	0.0612 ± 0.0078^∗∗^	0.0305 ± 0.0086	0.0349 ± 0.0060
*Prevotella*	0.0507 ± 0.0300	0.0507 ± 0.0473	0.0183 ± 0.0249
*Treponema*	0.0221 ± 0.0156	0.0079 ± 0.0081	0.0380 ± 0.0364
*Roseburia*	0.0389 ± 0.0345^∗^	0.0133 ± 0.0037	0.0036 ± 0.0024
*Gemmiger*	0.0197 ± 0.0090^∗∗^	0.0204 ± 0.0117^∗∗^	0.0025 ± 0.0008
*Ruminococcus*	0.0163 ± 0.0054^∗∗^	0.0089 ± 0.0031	0.0072 ± 0.0013
*Clostridiaceae*-Clostridium	0.0097 ± 0.0064	0.0095 ± 0.0039	0.0094 ± 0.0042
Others	0.5134 ± 0.0554	0.4696 ± 0.0869	0.4994 ± 0.1039

Note: TM stands for 60-day group, FM stands for 120-day group, SM stands for 180-day group; compared with SM ^∗^*P* < 0.05 and ^∗∗^*P* < 0.01.

## Data Availability

The original sequence obtained in this study has been submitted to the NCBI Sequence Read Archive (accession number is SRP: PRJNA795214, htttp://http://www.ncbi.nlm.nih.gov/).
